RETRACTED

# LRP6 Knockdown Ameliorates Insulin Resistance via Modulation of Autophagy by Regulating GSK3β Signaling in Human LO2 Hepatocytes

**DOI:** 10.3389/fendo.2019.00073

**Published:** 2019-02-12

**Authors:** Lei Li, Jing Xue, Jipeng Wan, Qian Zhou, Shan Wang, Yu Zhou, Heyong Zhao, Xietong Wang

**Affiliations:** ^1^Department of Obstetrics and Gynaecology, Shandong Provincial Hospital Affiliated to Shandong University, Jinan, China; ^2^Department of Obstetrics and Gynecology, The First Affiliated Hospital of Chongqing Medical University, Chongqing, China; ^3^Maternal and Child Health Care of Shandong Province, Jinan, China; ^4^Key Laboratory of Birth Regulation and Control Technology of National Health and Family Planning Commission of China, Jinan, China

**Keywords:** LRP6, insulin resistance, autophagy, GSK3β, hepatocytes

## Abstract

Recent studies suggest that autophagy is highly involved in insulin resistance (IR). Inhibition of the PI3K/AKT/mTOR signaling pathway induces autophagy activation. Additionally, depletion of LRP6 has been shown to increase insulin sensitivity but its mechanism is still not clear. We hypothesized that LRP6 contributes to IR by regulating mTOR mediated autophagy through GSK3β in hepatocytes. LO2 hepatocytes were treated with palmitate (PA) and insulin to induced IR. Levels of LRP6 mRNA and protein expression were measured by real time-PCR and western blot analysis. LRP6 knock down was achieved by adenovirus mediated Si-LRP6 expression and its roles in IR, glucose, GSK3β, mTOR signaling, and autophagy were explored. Finally, GSK3β was overexpressed and its involvement in autophagy and IR was examined. We found that PA treatment led to a reduced glucose uptake and IR in hepatocytes, which was accompanied by an upregulation of LRP6 expression. Knocking down of LRP6 enhanced glucose uptake and insulin sensitivity in PA treated cells, probably through increasing GSK3b activity. Overexpression of GSK3b mimicked LRP6 reduction by enhancing autophagy and ameliorating IR. Our study revealed a significant molecular mechanism connecting LRP6 to insulin sensitivity through GSK3β-mTOR mediated autophagy.

## Introduction

Insulin resistance (IR) plays a major role in the pathogenesis of several metabolic disorders, including type 2 diabetes, obesity, and hyperlipidemia. Although reduced physical activity and increased food, especially fat consumption, have been shown to contribute to IR, IR is a complicated condition with its exact mechanism still yet to be clarified (1, 2). Recently, accumulating evidence has pointed autophagy as an important player in the development of IR.

Autophagy is an important cellular process, responsible for removing intracellular debris and protein turnover (3). It is usually activated in stressed status such as starvation (4). In obese mice, IR is associated with downregulation of autophagy in the liver (5). Restoring autophagy enhances glucose tolerance and insulin sensitivity in obese mice. Increasing physical activity is associated with increased basal autophagy that improves glucose handling in diet-induced obese mice (6–8).

RETRACTED

Mammalian target of rapamycin (mTOR), a protein whose activity is largely dependent on the nutrient availability such as amino acid and glucose, is a negative regulator of autophagy (9). mTOR is activated by the PI3K-Akt pathway which is negatively regulated by GSK3β. mTOR phosphorylates key components such as Atg13 in the autophagy machinery. Inhibition of mTOR by rapamycin or nutrient starvation dephosphorylates Atg13 in mammalian cells, leading to induction of autophagy, accompanied by upregulation of Beclin 1 and LC3 II/I (10, 11).

A co-receptor of Wnt/β-catenin signaling pathway, low-density-lipoprotein-related protein 6 (LRP6) is involved in insulin resistance. Mice heterozygous for LRP6 are less prone to diet-induced obesity and are protected from insulin resistance (12). However, the detailed mechanism underlying this regulation is not clearly characterized. Previously, LRP6 has been shown to attenuate GSK3β activity (13). Although a link between LRP and autophagy has not been explored before, it is possible that LRP6 could potentially regulate mTOR signaling through modulating GSK3β activity, which may then negatively impact autophagy.

Palmitate (PA) is a saturated fatty acid that induces IR in various scenarios, including hepatocytes, although the molecular mechanism remains elusive (14). We hypothesized that PA treatment leads to differentiated expression of LRP6 that alters the activity of GSK3β and contributes to enhanced autophagy through mTOR in hepatocytes. In this current study, we explored the functions of LRP6 and GSK3β in PA induced IR in LO2 hepatocytes. Our finding revealed a significant molecular mechanism linking the function of LRP6 to IR through autophagy.

## Materials and Methods

### Cell Culture and Drug Treatment

LO2 hepatocytes were acquired from American Type Culture Collection (ATCC, Manassas, VA) and maintained according to standard procedure in high glucose Dulbecco's modified eagle medium (DMEM) supplemented with 10% fetal bovine serum, 100,000 U/L penicillin and 100 mg/L streptomycin. For palmitate (PA) and insulin treatment, cells were first cultured in 100 mm dishes to 80–85% confluence, washed with PBS three times, and then incubated in serum-free DMEM with 250 μM PA dissolved in ethanol and complexed to BSA at a 2:1 molar ratio for 24 h. Cells were then washed with PBS for three times and incubated in the absence or presence of 0.1 μM insulin for 10 min. An equivalent volume of ethanol added to 2% fatty-acid free BSA-DMEM was used as control treatment.

RETRACTED

### Western Blot Analysis

Cells were harvested and homogenized with RIPA buffer (50 mM Tris pH 8.0, 150 mM NaCl, 1% NP-40, 5 mM EDTA, 0.5% sodium deoxycholate, 0.1% SDS) supplemented with protease inhibitors and phosphatase inhibitors (Sigma, St. Louis, MO). Lysates with an equivalent amount of proteins were analyzed by Western blot using the following antibodies: anti-phospho-IRS1-S307, anti-IRS1, anti-phospho-AKT-Thr308, anti-AKT, anti-LRP6, anti-Beclin-1, anti-LC3, anti-phospho-GSK3β-Ser9, anti-GSK3β, and anti-β-actin. Antibodies were purchased from Abcam (Cambridge, MA, USA) unless it was specified. Western blot was quantified by densitometry using ImageQuant TL 1D v8.1 software (GE Healthcare Life Sciences, Little Chalfont, Buckinghamshire, United Kingdom). Data were normalized to control treatment.

### 2-NBDG Assay

2-NBDG assay was performed to assess glucose uptake in cells as previously described (15). Briefly, LO2 hepatocytes were first treated with control or 250 μM PA for 24 h and washed with PBS. Cells were then incubated in DMEM supplemented with 1 g/L glucose and 2% fatty acid free BSA for 3 h before being treated with or without 0.1 μM insulin for 10 min. After washing with Krebs buffer containing 0.5% BSA, cells were treated with 150 μg/ml 2-[*N*-(7-nitrobenz-2-oxa-1,3-diazol-4-yl) amino]-2-deoxyglucose (2-NBDG), a fluorescent 2-deoxygluocose glucose analog (Cayman Chemicals, Arbor, MI, USA) for 40 min. A microplate reader (Perkin Elmer VictorX4, Waltham, MA, USA) was then used to measure the fluorescent signal representing the amount of 2-NBDG uptake at a excitation wavelength of 485 nm and emission wavelength of 535 nm.

### Real Time-PCR (RT-PCR)

*Lrp6* mRNA levels were assessed by real time-PCR. Total RNA was prepared with TRIzol®RNA Isolation Reagents (company, catalog number). The same amount of RNA was used to synthesize cDNA through iScript™ cDNA Synthesis Kit (Life Technology, Pleasanton, CA, USA). RT-PCR was performed using SsoAdvanced™Universal SYBR®Green Supermix. Primers for Lrp6 are: 5′-CACTTACTTCCCTGCAATTTTGAACC-3′, and 5′-TGGCCTGTAGCTGTATGACCTATG -3′. *Lrp6* mRNA levels were normalized to control treatment.

### Recombinant Adenovirus Preparation and Infection

Expression vectors for recombinant adenovirus were constructed according to the Gateway cloning system (Invitrogen, Carlsbad, CA, USA) as previously described (16). Briefly, Si-LRP6, GFP-LC3, GSK3β were cloned into the pAD/CMB/V5-DEST vector and packaged by ViraPower Adenoviral expression system (Invitrogen, Carlsbad, CA, USA). LO2 hepatocytes were infected with adenoviruses that express Si-LRP6, GFP-LC3 or GSK3β at multiplicity of infection of 100 and harvested for further analysis after 48 h of infection.

RETRACTED

### GSK3β Activity Assay

GSK3β activity was assessed by GSK3 activity assay kit (Sigma, CS0990) according to manufacturer's instruction as described previously (17). Briefly, GSK3β in LO2 hepatocytes was immunoprecipitated with an anti-GSK3β antibody bound protein A/G affinity gel and incubated with γ-^32^P-ATP. GSK3β activity was measured by the incorporated ^32^P.

### Statistical Analysis

Data were represented as mean +/– SEM. Two-tailed unpaired *t*-test with equal variance was performed to determine the statistical difference between two groups. Significance was set at *p*-value <0.05.

## Results

### PA Disrupts Insulin Signaling and Blocks Glucose Uptake in LO2 Hepatocytes

We first investigated the effects of PA treatment on insulin signaling and glucose uptake in LO2 hepatocytes. We found that PA treatment alone significantly reduced the levels of phosphorylated IRS1 (p-IRS1) and AKT (p-AKT) compared to the control treatment (Figures 1A,B). Additionally, it also suppressed insulin induced upregulation of p-IRS1 and p-AKT. These results indicate that PA treatment leads to insulin resistance in LO2 hepatocytes. To further confirm this observation, we examined glucose uptake by 2-NBDG assay. We found that insulin significantly increased glucose uptake which was blocked by PA treatment (Figure 1C). In fact, PA treatment alone significantly reduced glucose uptake compared to that of control treatment.

**Figure 1:** PA treatment lead to IR and impaired glucose uptake in LO2 hepatocytes. **(A)** Insulin signaling was disrupted in PA treated LO2 hepatocytes. LO2 hepatocytes were treated with control or PA in the presence or absence of insulin. Cell lysates were processed for analysis by western blot using indicated antibodies. **(B)** Quantification of western blot analysis. Values were normalized to control treatment for each quantification. ^*^p < 0.05 vs. control-insulin group; #*p* < 0.05 vs. control + insulin group (*n* = 6). **(C)** Glucose uptake was assessed by 2-NBDG assay in LO2 hepatocytes. ^*^p < 0.05 vs. Control – insulin group, #*p* < 0.01 vs. Control + insulin group (*n* = 6).

### PA Treatment Upregulates LRP6 Expression

Since LRP6 has previously been shown to regulate insulin sensitivity (12), we hypothesized that PA induced insulin resistance through LRP6. To test this hypothesis, we examined the mRNA and protein levels of LRP6 in LO2 hepatocytes treated with PA. We found that while insulin slightly increased both mRNA and protein levels of LRP6, PA led to a substantial upregulation of these levels following 24 h treatment (Figures 2A,B).

RETRACTED

**Figure 2:** PA treatment increased LRP6 mRNA and protein expression in LO2 hepatocytes. LO2 hepatocytes were treated with control or PA in the presence or absence of insulin. **(A)** LRP6 mRNA levels were assessed by RT-PCR. **(B)** Western blot analysis of LRP6 protein expression in LO2 hepatocytes receiving indicated treatment. Data were normalized to control treatment in the absence of insulin. ^*^p < 0.05 vs. untreated control, #*p* < 0.05 vs. control+insulin (*n* = 6).

### LRP6 Knock Down Suppresses PA Induced Insulin Resistance

To determine if PA induced insulin resistance is indeed through upregulated LRP6, we investigated whether insulin resistance could be reversed by suppressing LRP6 expression. We knocked down LRP6 by adenovirus mediated Si-LRP6 expression and confirmed reduction of LRP6 protein in LO2 hepatocytes (Figure 3A). We found that LRP6 knock down significantly enhanced the insulin signaling pathway in the absence of PA treatment (Figures 3B,C). Additionally, LRP6 knock down also blocked PA-induced insulin resistance by increasing p-IRS1 and p-AKT levels. We further examined glucose uptake and found that LRP6 knock down significantly improved 2-NBDG uptake in the presence of PA treatment (Figure 3D).

**Figure 3:** Knock down of LRP6 attenuated PA-induced IR in LO2 hepatocytes. LO2 hepatocytes were infected with Ad-Si-LRP6 to knock down LRP6 protein expression. **(A)** LRP6 protein expression was reduced upon Ad-Si-LRP6 infection. ^*^p < 0.05 vs. control (*n* = 6). **(B)** Western blot analysis of insulin signal pathway following LRP6 knock down. **(C)** Quantification of western blot results. Data were normalized to control treatment for each protein. ^*^p < 0.05 vs. no-PA treatment control; #*p* < 0.05 vs. PA treatment group (*n* = 6). **(D)** LRP6 knock down enhanced glucose uptake in PA treated LO2 hepatocytes in the presence of insulin. ^*^p < 0.05 vs. no-insulin stimulated control; #*p* < 0.05 vs. PA treatment group (*n* = 6).

### LRP6 Knock Down Activates Autophagy in the Presence of PA Treatment

Since increasing autophagy has resulted in alleviating insulin resistance in hepatocytes, we investigated whether the induction of LRP6 expression after PA treatment was involved in regulating autophagy. We found that PA treatment significantly suppressed autophagy as indicated by reduced expression of autophagy markers Beclin-1 and LC3II/I (Figures 4A,B). Knocking down LRP6 significantly increased Beclin-1 and LC3II/I protein expression in the presence of PA treatment. Furthermore, we also examined autophagosomes by expressing LC3-GFP. We found that LC3-GFP autophagosome formation was abolished by PA treatment and reversed by knocking down LRP6 (Figures 4C,D). These results indicate that LRP6 downregulation attenuates insulin resistance by activating autophagy.

RETRACTED

**Figure 4:** Knock down of LRP improved insulin sensitivity through activation of autophagy in LO2 hepatocytes. **(A,B)** Western blot analysis **(A)** and quantification **(B)** showing that LRP6 knock down induced autophagy activation in LO2 hepatocytes (*n* = 6). **(C,D)** Representative images and statistical data of LO2 hepatocytes expressing GFP-LC3 via adenovirus infection upon on control, PA and/or Ad-Si-LRP6 treatment. ^*^p < 0.05 vs. no-PA treatment group; #*p* < 0.05 vs. PA treatment group.

### LRP6 Knock Down Induces Autophagy Through Modulating GSK3β Activity

Finally, we investigated GSK3β and mTOR signaling in PA treated LO2 hepatocytes. We found that PA treatment significantly reduced phosphorylated GSK3β (p-GSK3β) levels in the presence of insulin. LRP6 knock down increased the level of GSK3β, comparable to control treatment. Interestingly, we found that PA treatment suppressed mTOR phosphorylation (p-mTOR) (Figure 5A). In fact, LRP6 knock down further reduced p-mTOR levels after PA treatment. We asked whether LRP6 knock down induced GSK3β activation independent on phosphorylation. We examined GSK3β activity and found that PA treatment inhibited GSK3β activation. LRP6 knock out significantly enhanced GSK3β activity (Figure 5B).

**Figure 5:** GSK3β activation was involved in mediating the effects of LRP6 knock down on autophagy and insulin signaling. **(A)** LRP6 knock down inhibited mTOR in LO2 hepatocytes as shown by western blot analysis and quantifications of indicated proteins in the bar graph. ^*^p < 0.05 vs. no-PA treatment group; #*p* < 0.05 vs. PA treatment group (*n* = 6). **(B)** LRP6 activated GSK3β independent of inhibitory phosphorylation. ^*^p < 0.05 vs. no-PA treatment group; #p < 0.05 vs. PA treatment group (*n* = 6). **(C)** Overexpression of GSK3β activated autophagy in LO2 hepatocytes. Protein quantification was shown in the bar graph. ^*^p < 0.05 vs. control group; #*p* < 0.05 vs. PA treatment group (*n* = 6). **(D)** Overexpression of GSK3β attenuated insulin signal pathway disruption induced by PA treatment as shown by western blot analysis and quantifications of indicated proteins in the bar graph. ^*^p < 0.05 vs. control group; #*p* < 0.05 vs. PA treatment group (*n* = 6).

We then overexpressed GSK3β in LO2 hepatocytes and examined the effects on autophagy and insulin signaling. We found that GSK3β overexpression enhanced autophagy as indicated by increased levels of Beclin-1 and LC3 II/I in the presence of PA compared to that of PA treatment alone (Figure 5C). Additionally, we also found that GSK3β overexpression alleviated PA induced insulin resistance by upregulating p-IRS1 and p-AKT (Figure 5D).

RETRACTED

## Discussion

Understanding the molecular mechanism underlying insulin resistance will have significant implications in the development of therapeutic strategies against multiple metabolic disorders including type II diabetes. In the current study, we investigated the signaling pathway connecting LRP6 to IR in hepatocytes. We first confirmed that PA treatment in hepatocytes induced IR by suppressing glucose uptake and phosphorylation of key components in insulin signaling including IRS1 and AKT. We found that LRP6 expression was substantially upregulated as a result of PA treatment and knock down of LRP6 restored IRS1 and AKT phosphorylation and glucose uptake. This correlates with an induction of autophagy which was suppressed by PA treatment alone. Importantly, we found that LRP6 regulated insulin sensitivity through GSK3β and knock down of LRP6 enhanced GSK3β activity. Consistent with this observation, we found that overexpression of GSK3β in PA treated hepatocytes also restored autophagy induction and insulin signaling, as indicated by rescued IRS1 and AKT phosphorylation. To our knowledge, this is the first study linking LRP6 function to fat induced insulin resistance through autophagy.

Wnt signaling has been implicated in the pathogenesis of metabolic disorders including type 2 diabetes (18, 19). A single missense mutation in LRP6 that impairs Wnt signaling was identified in patients with metabolic syndrome (19). A previous study using heterozygous mice showed that LRP6 was involved in insulin resistance (12). Mice that were missing one copy of the LRP6 gene were protected from high fat induced obesity and insulin resistance, indicating that LRP6 may be negatively correlated with insulin sensitivity. However, it is not clear whether fat induced insulin resistance involves differential regulation of LRP6 expression. Our study revealed that the saturated fatty acid PA significantly enhanced both LRP6 mRNA and protein levels. Consistent with the mouse LRP6 heterozygous study, our results using adenovirus mediated LRP6 knock down strategy indicated that modulating LRP6 levels may be sufficient to overcome insulin resistance in human hepatocytes. Although not frequent, a loss-of-function mutation (*LRP6*_*R*611*C*_) has been identified in some patients with impaired insulin sensitivity (20). This study together with our finding suggest that a low expression level of LRP6 with normal function is both required and sufficient to maintain insulin reactivity.

RETRACTED

A loss-of-function mutation of LRP6 resulted in a reduction of GSK3β phosphorylation in response to insulin stimulation, as compared to cells with wild type LRP6 (20). Interestingly, our study also found enhanced GSK3β phosphorylation in LRP6 knock down hepatocytes. However, we observed an increased GSK3β activity independent on phosphorylation, which was accompanied by reduced mTOR activation. mTOR complex 1 (mTORC1) activity was reduced in LRP6 heterozygous mice and increased in cells carrying a LRP6 loss-of-function mutation (12, 20, 21). mTOR activation prevents apoptosis while inhibition of mTOR signaling is necessary to activate autophagy to remove intracellular debris (22). Interestingly, a link between LRP6 and autophagy has not been established prior to our study.

Autophagy is an important cellular process that protects cells by removing unnecessary proteins. Deletion of a critical autophagy gene Atg7 in the liver leads to accumulation of hepatic fat, indicating that autophagy is involved in fat metabolism (23). Recent accumulating evidence has identified autophagy as an important player in insulin signaling and glucose metabolism (24). Autophagy has been shown to be important for the maintenance of the normal function of insulin targeting tissues such as the liver, and the homeostasis of pancreatic β-cells. β-cell dysfunction is associated with impaired autophagy (25). However, consistent results have not been reached. Some studies showed that defective autophagy promoted insulin resistance while some reports pointed to the opposite, showing that autophagy deficiency actually protects from insulin resistance (5, 26, 27). We believe the function of autophagy in insulin resistance may be cell type specific. Consistent with the study in liver (5), we found that PA treatment-induced insulin resistance was accompanied by suppressed autophagy in hepatocytes. Importantly, we found that knock down of LRP6 rescued autophagy in PA treated hepatocytes which is in line with a function of autophagy in maintaining insulin sensitivity.

As previously stated, our results indicate that LRP6 regulates GSK3β activity. Since GSK3β is a negative regulator of mTOR signaling, we further explored the relation between GSK3β and autophagy in PA treated hepatocytes. We found that adenovirus-mediated GSK3β overexpression not only restored the levels of autophagy related proteins back to control status, but also enhanced insulin sensitivity. Thus, our results suggest that enhancing GSK3β expression alone is also sufficient to suppress fat induced insulin resistance in hepatocytes.

RETRACTED

Although beyond the scope of our current study, further detailed study is necessary to characterize the potential adverse effects when developing therapeutic strategies. Another limitation is that this study was focused on one cell type. One future direction for this research will be to characterize this signaling pathway in more cell types. Nevertheless, our study revealed a significant link among LRP6, GSK3β, autophagy, and fat induced insulin resistance.

## Conclusion

In summary, our findings suggest that fat induced insulin resistance may be caused by enhanced LRP6 expression, which leads to suppressed autophagy. Our results point to GSK3β being a bridge connecting LRP6 to insulin resistance. Since modulating LRP6 and GSK3β expression levels is sufficient to alter the status of insulin sensitivity in hepatocytes, altering LRP6 and GSK3β expression may represent a potential therapeutic strategy for insulin resistance associated metabolism disorders.

## Author Contributions

LL, JX, JW, QZ, SW, and YZ, collected and analyzed the data. HZ and XW designed the study and wrote the manuscript.

### Conflict of Interest Statement

The authors declare that the research was conducted in the absence of any commercial or financial relationships that could be construed as a potential conflict of interest.
